The article "Novel Hybrid Gels Made of High and Low Molecular Weight Hyaluronic Acid Induce Proliferation and Reduce Inflammation in an Osteoarthritis In Vitro Model Based on Human Synoviocytes and Chondrocytes" was retracted in 2022. Reasons: duplicated images; unreliable data; concerns about the data.

# Novel Hybrid Gels Made of High and Low Molecular Weight Hyaluronic Acid Induce Proliferation and Reduce Inflammation in an Osteoarthritis* In Vitro* Model Based on Human Synoviocytes and Chondrocytes

**DOI:** 10.1155/2019/4328219

**Published:** 2019-04-23

**Authors:** Antonietta Stellavato, Valentina Vassallo, Annalisa La Gatta, Anna Virginia Adriana Pirozzi, Mario De Rosa, Giovanni Balato, Alessio D'Addona, Virginia Tirino, Carlo Ruosi, Chiara Schiraldi

**Affiliations:** ^1^Department of Experimental Medicine, Section of Biotechnology, Medical Histology and Molecular Biology, University of Campania “Luigi Vanvitelli”, Naples, Italy; ^2^School of Medicine and Surgery “Federico II” of Naples, Department of Public Health, A.O.U. Federico II of Naples, Via S. Pansini, 80131 Naples, Italy

## Abstract

High molecular weight hyaluronan (H-HA) has a pivotal role in the maintenance of normal functions of synovial fluid and structure of the articular joint, but it has been shown that its concentration is reduced in patients affected by degenerative cartilage diseases, such as osteoarthritis (OA). The aim of this study was to investigate the anti-inflammatory effects and properties of hybrid cooperative complexes based on high and low molecular weight hyaluronan (HCC) compared to H-HA on human primary cells derived by pathological joints. In addition, the rheological behavior of HCC was evaluated in order to define their potential as viscosupplement gel in degenerated joints. The experiments were performed using an* in vitro* model of OA based on human chondrocytes and synoviocytes isolated from degenerated joints of patients hospitalized for surgical replacement. In order to assess the anti-inflammatory effects of HCC, we evaluated NF-kB, COMP-2, IL-6, and IL-8 as specific markers at the transcriptional and/or protein level. Moreover, the proliferative properties of HCC were assessed using time lapse video microscopy. We showed that chondrocytes and synoviocytes clearly presented an altered cytokine profile compatible with a severe ongoing inflammation status. H-HA and, above all, HCC significantly reduced levels of the specific biomarkers evaluated and improved cartilage healing. The rheological profile indicated HCC suitability for intra-articular injection in joint diseases. HCC viscoelastic properties and the protective/anti-inflammatory effect on human chondrocytes and synoviocytes suggest the novel HCC-based gels as a valid support for OA management.

## 1. Introduction

Osteoarthritis (OA) is a progressive disease of the synovial joints that causes pain and limitation of function worsening the quality of life. Knee is the most common OA localization, affecting more than 250 million people worldwide with consequent social and economic burden [1]. An estimated 10% of men and 18% of women over 60 years of age suffer of this onset [2, 3]. It has been evaluated that in developed countries the cost for health care system may reach up to 25% of gross domestic product [4]. Traditionally, OA conservative treatment consists of pain management (pain therapy, intra-articular injections, and anti-inflammatory drugs), but joint replacement is considered the definitive treatment for end-stage disease [1]. Several studies have focused on identifying potential modulators of osteoarthritic symptomatology [2]. In particular, regulation of the inflammatory response in synovial fibroblasts is considered a useful therapeutic strategy against both the symptoms and the progression of OA pathology [5]. Articular cartilage is a connective tissue composed of chondrocytes, a type of cell surrounded by a viscous extracellular matrix (ECM). Chondrocytes represent about 2-5% of cartilage tissue, while the ECM is composed of water (about 75% of the total weight), proteoglycans and glycosaminoglycans (20% of the total weight), specifically type II collagen fibers accounting for 5% of the total [6]. Synovial fluid plays an essential role in the lubrication of joints, and it is characterized by two types of cellular populations: type A synoviocytes (macrophage-like) and type B synoviocytes (fibroblast-like). The former derive by bone marrow and are totally differentiated [7, 8] while the latter are of mesenchymal origin and display many characteristics of fibroblasts and produce several proteases during the process of cartilage damage [8–10]. It has been shown that the first population disappears during* in vitro* incubation while type B synoviocytes continue to grow in clusters. Type B synoviocytes are involved in controlling the composition of the synovial fluid. Normally, they produce collagen (in particular collagen type IV), fibronectin, hyaluronic acid, and several proteoglycans into joint cavities [11]. Recent studies about OA have shown that the proinflammatory protein nuclear factor kappa-light-chain-enhancer of activated B cells (NF-kB) plays a key role during the development and progression of cartilage diseases [12, 13]. Finally, chondrocytes also produce cartilage oligomeric matrix protein (COMP), which is involved in the reconstitution of articular cartilage after damage, and, in this context, its overexpression was shown to be related to degenerative conditions, such as OA [3, 14]. However, COMP is produced by various types of mesenchymal cells, including synoviocytes. For this reason, this is considered a key marker of cartilage degeneration, and its presence in synovial fluid may help in the evaluation of pathology progression. Furthermore, synovia is a tissue largely involved in articular pathologies [15]. It has been proved that, in the synovial fluid of patients with OA, there is an increase of proinflammation cytokines [13, 16, 17]. Nowadays, OA approaches are based on (a) physical and occupational therapies; (b) pharmacological treatments for pain management such as paracetamol, nonstreoidal anti-inflammatory drugs (NSAID), opioid and corticosteroids injections; (c) surgical procedures such as arthroscopy, microfracture, or total joint replacement in severe OA conditions [18]. Injections of hyaluronan gels can reduce the inflammation state, provide pain relief, and give a viscosupplementation effect in the joints [19, 20]. HA increases the proliferation of chondrocytes and reduces the expression of proinflammation markers, but linear HA turnover* in vivo* is often fastened in pathological conditions [19, 21]. To date, the possibilities of slowing down this phenomenon have been related to either chemical modification through cross-linking agents or biophysical interactions to obtain hybrid complexes. Specifically, hybrid complexes are based on high and low molecular weight of pharma-grade HA, and their properties have been tested in several* in vitro* cellular models [19, 22–25]. The aim of this study was to investigate the anti-inflammatory effect and properties of HCC compared to H-HA in an OA* in vitro* model based on human cells derived from degenerated knee cartilage and the corresponding synovial fluid.* In vitro* models are useful to shade light on the biochemical and cellular mechanisms beyond thus, tissue repair.  Figure 1 is a schematic representation of the signaling pathway investigated with related techniques.

## 2. Materials and Methods

### 2.1. Hyaluronic Acid-Based Gels

High molecular weight (H-HA; MW 1400±200 kDa) and low molecular weight (MW 100±20 kDa) hyaluronic acids were provided by Altergon (Altergon s.r.l., Italy). These are fermentative HA of high purity (SHYALT®) derived from* Streptococcus equi* ssp.* equi*, extensively purified at pharmaceutical grade (e.g., purity >95%, water content <10%, Endotoxin Units, EU/mg <0.05, and very low metal contents). pH and osmolality were measured in order to perform experiments in physiological conditions (i.e., pH 7.0±0.1; osmolality 300 mOsm). H-HA was dissolved in Phosphate-Buffered Saline (PBS, pH 7.2, Lonza), at a concentration of 16 g/L; the resulting solution was thermally treated following the same protocol assessed to obtain hybrid cooperative complexes (HCC) [27]. HCC, commercialized as Sinovial-HL®, contain 16 mg H-HA and 16 mg L-HA in 1 mL volume and were provided in prefilled syringes. Sinovial-HL® was provided for this study by IBSA Farmaceutici. HCC were diluted in PBS in order to have an intermediate concentration of 16 g/L. Finally, all the solutions were diluted at a concentration of 3.2 g/L in the culture medium (DMEM Dulbecco's modified Eagle's medium, Gibco, Invitrogen).

### 2.2. Rheological Studies

Measurements were carried out using a Physica MCR301 oscillatory rheometer (Anton Paar OS, Germany). Flow curves were obtained using coaxial cylinders geometry (CC27-SN7969; measuring cup diameter/measuring bob diameter: 1.0847 according to ISO 3219; gap length 39.984 mm; sample volume 19.00 mL). Specifically, the dynamic viscosity of the samples was registered as a function of shear rate (0.001–300 s^−1^) at 25°C, 50 measuring points. Strain and frequency sweep tests were performed using a CP 50-1 geometry (cone diameter 49.968mm, cone angle 0.994°, truncation 100*µ*m). Strain sweep tests were carried out at 1 Hz frequency over a strain amplitude range of 0.01–100%, at 37°C; 50 measuring points were acquired with no time setting. Oscillation frequency sweep tests were then carried out over a frequency range of 0.1–10 Hz; at a constant strain selected within the linear viscoelastic range (1%), 20 measuring points/dec were acquired at 37°C. The values of the moduli at 0.5 and 2.5 Hz (physiological walking and running frequency) were derived.

### 2.3. Assessment of Cytokines Presence in Osteoarthritic Synovial Fluids by a Bio-Plex Cytokine Assay

The synovial fluids isolated from five patients and obtained during the surgical procedure were centrifuged (1500 rpm, 7 min), and the supernatants were stored at -80°C. A human cytokines assay (Bio-Rad Laboratories s.r.l., Milan, Italy), including Granulocyte-Macrophage Colony-Stimulating Factor (GM-CSF), Interferon gamma (INF-*γ*), Interleukin-2 (IL-2), Interleukin-4 (IL-4), Interleukin-6 (IL-6), Interleukin-8 (IL-8), and Tumor Necrosis Factor-alpha (TNF-*α*), was performed. A multiplex assay was carried out according to the manufacturer's instructions using a Bio-Plex array reader (Luminex, Austin, TX). Cytokines concentrations (pg/mL) were evaluated by a standard curve according to the manufacturer's protocol. The multiplex analyses were performed in triplicate wells for each experimental point of two separate experiments.

### 2.4. Isolation and Culture of Human Chondrocytes and Synoviocytes

The knee cartilage and synovium samples were obtained from five patients affected by OA who underwent a total joint replacement at the Orthopedics and Traumatology Department of the University Federico II of Naples. All patients gave an informed consent, and all the procedures were allowed by the Internal Ethical Committee. We received two different specimens of cartilage from the same knee; one sample of cartilage was harvested from a piece of intact cartilaginous tissue of the knee, considered a healthy part and used as the control (healthy control; H-CTRL). The other sample was harvested from an extensively damaged cartilage tissue of the same knee (pathological control; P-CTRL). Primary cell isolation was obtained with a slight modification of the specific protocol previously published [19]. Specifically, cartilage tissue was minced into small pieces and digested in a solution composed of collagenase type I at 3 mg/mL (Gibco, Invitrogen, MA, USA), dispase at 4 mg/mL (Gibco, MA, Invitrogen) diluted in PBS, and Gentamycin 0.2 mg/mL (Hospira, IL, USA) at the temperature of 37°C on a shaking plate overnight. The cells were separated from undigested pieces through a sterile filter (70 *μ*m, Falcon) and the cellular suspension was centrifuged at 1500 rpm for 7 min (Eppendorf Centrifuge). The pellet was then washed with PBS, recentrifuged and resuspended in DMEM supplemented with Fetal Bovine Serum (FBS) (10% v/v) (Gibco, MA, Invitrogen), penicillin-streptomycin (1% v/v), and Amphotericin B (1% v/v) (Lonza, Basel, Switzerland). The cells were seeded in a 35 mm tissue culture well and maintained at 37°C in a humidified atmosphere with 5% v/v CO_2_, and the medium was changed every 48h. The synovial fluid samples were centrifuged, the supernatants were removed, the pellets were washed with PBS, and the cells were seeded following the same protocol used for the chondrocytes. The obtained synoviocytes cultures from synovial fluids isolates from OA patients and untreated cells (CTR) were indicated as UT-S in comparison to H-HA and HCC-treated cells.

### 2.5. Phenotypic Characterization of Articular Chondrocytes through Fluorescence-Activated Cell Sorting (FACS)

Chondrocytes were used at 2nd and 3rd passage, and their cellular phenotype was confirmed through the evaluation of specific antigens as previously reported. In particular, FACS analyses confirmed the cellular expression of type II collagen that was indicated as specific biomarker of chondrocyte phenotype [3, 19].

### 2.6. Phenotypic Characterization of Synoviocytes through FACS

After 3 weeks of culture, the cells were harvested with trypsin/EDTA 0.2 mg/mL, centrifuged (1500 rpm, 7 min), and the supernatant was removed. Finally, the pellet was resuspended in PBS and analyzed (passage 1) through FACS in order to evaluate specific cellular markers surface expression. The experimental protocols followed have been previously described [3, 19]. The synoviocytes used to perform the experiments were harvested between the 2nd and 4th passage. Each experiment was performed in triplicate wells for each experimental point.

### 2.7. Evaluation at Protein Level of COMP-2 and NF-kB through Western Blotting Analyses

After 3 weeks, the chondrocytes were harvested with trypsin/EDTA 0.2 mg/mL and reseeded into a 12-well tissue plate, 5.0 x 10^4^ cells/cm^2^ (passage 2). After 48h of treatment with H-HA (0.32% w/v) and HCC (0.32% w/v), western blotting (WB) analyses were performed as previously described [28]. The synoviocytes were also analyzed through WB after 96h of treatment. The use of the different treatment time for the two cell model is ascribed to the different growth rates; specifically synoviocytes are slower than chondrocytes. All the cells were lysed by a Radio-Immunoprecipitation Assay (RIPA buffer) (1x) (Cell Signaling Technology), protein concentrations were evaluated using the Bradford method, and 30 *μ*g of intracellular proteins were electrophoretically resolved on 10% SDS-PAGE. The separated proteins were transferred to a nitrocellulose membrane (GE, Amersham, UK), and it was blocked with 5% nonfat milk in Tris-buffered saline and 0.05% Tween-20 (TBST). Specifically, for NF-kB, nuclear protein extraction was used to analyze NF-kB protein activity related to nuclear translocation. Primary antibodies to detect COMP-2 (Abcam, Cambridge, UK) and NF-kB (Santa Cruz Biotechnology, CA, USA) were used at 1:500 dilutions and were incubated for 2h at room temperature (RT). After extensive washing with TBST, immunoreactive bands were detected by chemioluminescence using corresponding horseradish peroxidase-conjugated secondary antibodies (Santa Cruz Biotechnology, CA, USA), diluted 1:10000 for 1h at RT and reacted with an ECL system (Millipore). Protein levels were normalized with respect to the signal obtained with an anti-Actin antibody 1:500 dilution (Santa Cruz Biotechnology, CA, USA). The semiquantitative analysis of protein levels was carried out using the Gel Doc 2000 UV System according to the manufacturer's protocol. Western blotting analyses were performed on two separate SDS-PAGE and each experiment was performed in duplicate for each experimental point.

### 2.8. Assessment of Cytokines Secretion and Their Modulation in the Presence of Hyaluronan by a Bio-Plex Cytokine Assay

Also, the culture media of chondrocytes treated with H-HA (0.32% w/v) and HCC (0.32% w/v) for 48h were preserved at -80°C. A human cytokine assay (Bio-Rad Laboratories s.r.l., Milan, Italy) was performed as described in the previous, Section 2.3 of Materials and Methods.

### 2.9. Cell Proliferation Assay Performed on Synoviocytes in the Presence of Hyaluronan

The synoviocytes were harvested with trypsin/EDTA 0.2 mg/mL and reseeded into a 24-well tissue plate, 1.0 x 10^4^ cells/cm^2^ (passage 3). After 2h, the culture medium was removed and replaced either by fresh medium (pathological control untreated cells; UT-S), a medium containing H-HA (0.32% w/v), or HCC (0.32% w/v). The assay lasted 5 days; every day the cells were observed by an inverted microscope (Leica Microsystem) and photos were taken by a Nikon Camera. A double count of the cells was performed using the traditional Burker chamber and Image-Pro Plus 1.5 analysis software (Media Cybernetics) following the assayed procedure reported in the literature [29]. Each cell count was performed in duplicate wells for each experimental point.

### 2.10. Quantitative Gene Expression of IL-6 and IL-8 through qRT-PCR in Human Synoviocytes Isolated from Knee Synovial Fluid

The synoviocytes used for the proliferation assay were further employed to assess the mRNA expression of IL-6 and IL-8 after 24 and 48h of treatment with H-HA and HCC 0.32% w/v. Total RNA was isolated using TRIzol® Reagent (Invitrogen, Milan, Italy) as previously described. The RNA concentration of each sample was evaluated using a Nanodrop Instrument (Celbio, Milan, Italy) and 1 *µ*g of total RNA was reversely transcribed into cDNA with the Reverse Transcription System Kit (Promega, Milan, Italy) following the manufacturer's protocol. Finally, a quantitative Real-Time PCR was performed by the IQ™ SYBR® Green Supermix (Bio-Rad Laboratories, Milan, Italy); the primer sequences used for our gene analyses are reported in Table 1. The samples were analyzed in triplicate, and the mRNA expression of specific genes was normalized with respect to the glyceraldehyde-3-phosphate dehydrogenase (GAPDH) housekeeping gene [3]. The variations of gene expressions were evaluated through Livak's method 2^-ΔΔCt^ (ΔΔCt = difference of ΔCt between H-HA- or HCC-treated cells and control) using Bio-Rad iQ5 software (Bio-Rad, Milan, Laboratories).

### 2.11. Data Analysis

For all experiments performed, results are shown as mean ± standard deviation (SD). Statistical analysis was performed using Student's* t* test. Values were considered statistically significant when* p *values were less than 0.01 or 0.05.

## 3. Results

### 3.1. Rheological Measurements: Viscoelastic Behavior

The results of the rheological characterization of HCC are reported in Figure 2. The flow curve of the preparation (Figure 2(a)) indicates a pseudoplastic behavior, with a value of zero-shear viscosity equal to 12.1 Pa s. Viscosity remains constant within 0.3 s^−1^ shear rate and then reduces with a shear thinning ratio (*η*0.1/ *η*250) of about 13. The mechanical spectrum (Figure 2(b)) indicates an essential fluid behavior at low frequency values with G” exceeding G'. Both moduli increased in frequency with a faster G' increase until a crossover point registered at about 4Hz. At higher frequencies, the preparation exhibited an essential elastic behavior with G' exceeding G”. The G' values for HCC at 0.5 and 2.5 Hz frequency are 13.7 and 58.6 Pa, respectively.

### 3.2. Characterization of Synovial Fluids of Patients Affected by Osteoarthritis by Bio-Plex Cytokine Assay

A Bio-Plex cytokines assay was performed in order to evaluate the profile of human knee synovial fluid, extracted from patients undergoing surgical replacement for severe OA. The overall cytokine secretion pattern is reported in Figure 3. The results show that the samples analyzed presented a high content of IL-2, IL-6, and IL-8. The measured cytokines values are in fact significantly higher than the ones reported in literature as average values for synovial fluids of healthy donors (Figure 3) [17]. However, the concentration of TNF-*α* and GM-CSF were found to be low. IL-8 was the most expressed. This is in agreement with literature reports since it is produced by both chondrocytes and synoviocytes, which play an important role during the inflammation onset [30, 31].

### 3.3. *In Vitro* Phenotype Characterization of Human Articular Chondrocytes

According to data analyses previously reported, type II collagen was selected as specific chondrocyte biomarker [3, 19] in order to confirm the cellular phenotype (data reported in supplementary file (available here)).

### 3.4. FACS Characterization of Cultured Fibroblast-Like Synoviocytes

FACS analyses revealed that the population of cells isolated from human knee synovial fluid (at first passage of culture) was composed of type A synoviocytes, representing about 20.8% of the total population characterized by CD45^+^CD64^+^CD14^+^CD105^+^CD73^+^CD90^±^CD3^−^CD19^−^CD34^−^ phenotypes. In contrast, type B synoviocytes represented about 51.4% of the total cellular population characterized by CD105^+^CD73^+^CD90^+^CD45^−^CD64^−^CD14^−^CD3^−^CD19^−^CD34^−^ phenotypes (as reported in supplementary material). CD45^−^ and CD14^−^ are typical markers of monocyte-macrophage differentiation while CD90^+^, CD73^+^, and CD105^+^ are typical mesenchymal markers. Before their use for our experiments, it was confirmed that the majority of the cellular population was composed of type B synoviocytes,

### 3.5. Hyaluronan Anti-Inflammatory Activity through the Evaluation of NF-kB and COMP-2

Western blotting analyses revealed that, at baseline, the cells isolated from damaged cartilage (P-CTRL) showed high levels of the proinflammatory protein NF-kB and COMP-2 with respect to H-CTRL (p<0.01) (Figure 4(a)). After 48h of H-HA treatments, the expression of both markers analyzed decreased. In particular, H-HA reduced significantly (p<0.05) the expression level of NF-kB by about 30% with respect to P-CTRL. Besides, the anti-inflammatory effect of the HCC complexes was higher since it induced a 60% reduction of NF-kB expression (p<0.01) with respect to P-CTRL and p<0.05 with respect to H-HA (Figure 4(a)). Also, the expression of COMP-2 was about 40% lower in the cells treated with HCC (p<0.05) with respect to P-CTRL while H-HA cells reduced COMP-2 by about 15% (p<0.05) (Figure 4(a)). After 96h of treatment, the expression of NF-kB was reduced by about 35% in synoviocytes treated with HCC (p<0.05) in comparison with UT-S; the H-HA-treated cells did not seem to be affected (p<0.05) (Figure 4(b)). We also evaluated the expression levels of COMP-2. Its expression was slightly reduced by H-HA treatment with respect to UT-S; however, a superior reduction of about 25% of this biomarker was obtained by HCC treatment (Figure 4(b)).

### 3.6. Cytokines Level Quantification of Chondrocytes Using Bio-Plex Cytokine Assay

Bio-Plex was performed on culture media of chondrocytes. Data showed that all cytokines were upregulated in P-CTRL cell cultures with respect to H-CTRL (Figure 5). Specifically, GM-CSF, INF-*γ*, and TNF-*α*, (Figures 5(b), 5(d), and 5(e)) were significantly different (p<0.05). H-HA-treated samples showed a significant decrease of GM-CSF and TNF-*α* levels with respect to P-CTRL while HCC treatments showed marked beneficial effects in reducing all proinflammatory cytokine levels. Specifically, IL-6, IL-8, and INF-*γ* were reduced by about 1.32, 1.36, and 1.33 fold, respectively, with respect to the pathological control, TNF-*α* was reduced by 2.33 fold, and the GM-CSF reduction reached 3.47 fold. IL-2 and IL-4 quantifications were not reported because the relative absorbance values were below the detectable expression level with respect to Bio-Plex calibration curve.

### 3.7. Cell Viability and Proliferation Assay Performed on Human Synoviocytes

As shown by the growth curves (Figure 6(b)), HCC promoted cell proliferation faster than H-HA, which, as expected, improved cell viability with respect to the UT-S after 24h of treatment (Figure 6(a)). Our results showed that after 96h, HCC-treated cells increased by 72 ± 4% the number with respect to the initial condition. H-HA prompted a 61 ± 3% increase while UT-S obtained only a 52 ± 4% increment.

### 3.8. Specific Inflammatory Genes Analyses Using Quantitative Real-Time PCR (qRT-PCR) Performed on Synoviocytes

The qRT-PCR results reported in Figure 7(a) show that both H-HA and HCC significantly reduced the expression of IL-6 and IL-8 (p<0.05- p<0.01, respectively) with respect to the UT-S. However, at 24h, the reduction obtained by HCC of about 10-fold was significantly superior to the one obtained in H-HA treatment (~5-fold) for the 2 markers (p<0.05). Moreover, HCC further reduced significantly IL-6, also at 48h (Figure 7).

## 4. Discussion

It is well known that the reduction of the viscoelastic properties of the synovial fluid may accelerate joint degeneration. In particular, it has been shown that, in patients with OA, the properties of synovial fluid are altered and molecular weight and concentration of HA are reduced [32]. Thus, synovial cells lose their lubricant function and produce several types of cytokines, chemokines, and proteinases, which are responsible for the degradation of the extracellular matrix [33, 34]. In this context, viscosupplementation, based on the restoration of the viscoelastic features of synovial fluid through the intra-articular injections of suitable material, is currently one of the therapeutic strategies most used. Due to its viscoelastic properties, HA is the most-exploited material in existing pharmaceutical formulations and medical devices. The present research aimed at investigating the new HCC, based on high and low molecular weight HA, obtained through a patented procedure that may represent an innovation in OA management [21]. The rheological characterization of the HCC formulation (Figure 2) indicated a typical entangled network resembling those reported for healthy synovial fluid. The zero-shear viscosity and the dynamic moduli values are in agreement with the widely used HA-based intra-articular medical devices, thus predicting an appropriate response to stress conditions when injected [35–39]. Beside the viscoelastic properties, another crucial requirement is the injectability through fine bore needles to reduce pain during delivery [40]. In this respect, even if the HCC formulation is the highest concentrated one among commercial intra-articular injectables, it can be delivered using a 29-Gauge needle because of the HCC-specific viscosity features and shear thinning behavior (Figure 2(a)) [40–42]. Finally, HCC already proved to be highly resistant to hyaluronidase-catalyzed degradation with respect to linear HA supporting a prolonged viscosupplementation effect [42]. Beyond the biophysical reconstitution of synovial fluid, the main therapeutic targets are inflammation state and related pain [43]. In fact, it has been reported that synovial inflammation is a recurrent factor in OA, and this condition may be responsible for the disease progression [44–46]. However, chondrocytes may also contribute to inflammatory cytokines secretion into synovial fluids [13]. A few therapies are now suggested for OA treatment, but none of those leads to pathology remission or tissue regeneration. For these reasons, research has been concentrated on the development of new treatments for OA [47], mainly aiming at the modulation of the principal inflammatory mediators, such as cytokines [48–50]. In the present study, in addition to their well-known biophysical properties, we investigated the HA-based gels biological and biochemical features and Figure 1 sketches the OA signaling that we explored. Since their important role in OA* in vitro* models based on chondrocytes and synoviocytes are very useful for disease studies. In particular, several scientific reports described the use of* in vitro* models of this pathology obtained insulting chondrocytes and/or synoviocytes with IL-1*β* or IL-17 in order to mimic the OA catabolic and inflammatory process [2, 51] whereas our* in vitro* model is based on articular cells isolated from OA affected patients already presenting an ongoing inflammatory process. The study reported is, in this respect, better resembling actual/real* in vivo *conditions. It has been proved that the composition of healthy synovial fluids is different from, pathological samples, being the latter rich of cytokines, along with angiogenetic and growth factors [26]. Our data about cytokines expression in OA samples proved coherent with scientific reports [16, 17]; in fact, we assessed a high expression of the principal proinflammatory cytokines related to the pathology. In particular, according to Papalia and collaborators [26] we reported an over expression of IL-6 and TNF-*α*; furthermore, we found an upregulation for IL-8 and in agreement with Kjelgaard-Petersen and collaborators [48]. However, it has to be considered that here we present the average data of synovial fluid cytokines content only of five patients; thus, a larger sampling should be accomplished in the future to better investigate the key biomarkers to confirm the presented data. Inflammation balance is important for the cells survival, and it is well established that NF-kB is active in immune and inflammatory responses while COMP-2 is an important biomarker related to articular diseases. In agreement with numerous reported studies [52–54], those biomarkers are activated during inflammatory response. We demonstrated that HCC were more effective than H-HA gels in reducing these protein levels. A multiplex ELISA assay corroborated these results highlighting the anti-inflammatory effects of hyaluronan based treatments (Figure 5). Synovial cell populations were a preferred cell model in order to further explore cellular and molecular pathways related to OA [55]. These cells have genotypic mesenchymal features and show proliferating properties, thus being suitable for* in vitro* expansion [56]. The proliferation assay, as expected, proved an increase of synoviocytes cell growth in the presence of HCC in comparison to H-HA-treated cells and UT-S. Finally, Ahn and collaborators [30] reported that osteoarthritic synoviocytes release inflammatory cytokines contributing to the advancement of disease. In this study we showed that HCC and H-HA were able to reduce IL-6 and IL-8 expression at transcriptional level in this cellular type. Notwithstanding, more reliable data should be supported by experiments on a larger number of patients. However, we can be confident of the predicted positive clinical outcome since different* in vivo* studies have already been performed in order to demonstrate the beneficial effects of hybrid complexes beyond the efficacy of HA-based viscosupplementation therapy [7, 57]. For this reason, there exists a solid basis to hypothesize that HCC could become a more performing support as a medical device for the treatment of OA symptomatology.

## 5. Conclusions

The results of the rheological characterization indicate that HCC may provide suitable viscosupplementation combined with proper injectability. HCC had an anti-inflammatory effect on human chondrocytes and synoviocytes when isolated from pathological knee joints. The results of all experiments performed showed that HCC were more effective than linear H-HA. HCC reduced IL-6 and IL-8 gene expression levels as well as COMP-2 and NF-kB protein expression in both cells types populating human joints. Also, HCC gels prompted synoviocytes proliferation. Future* in vivo* models will better validate HCC as a therapeutic tool for the management of OA.

## Figures and Tables

**Figure 1:** Schematic resume of signaling investigated with related techniques used; in particular, synovial fluid and type B chondrocytes and synoviocytes have been objects of our studies. Gene expression and protein production were analyzed to assess the inflammation status in OA joints and then in derived cell populations.

**Figure 2:** HCC rheological characterization. (a) HCC dynamic viscosity as a function of the shear rate. (b) Dynamic Moduli for HCC as a function of the frequency.

**Figure 3:** Analysis of synovial fluids of four patients affected by OA by the Pro-Human Cytokine Multiplex Assay. The levels of the following cytokines were analyzed; GM-CSF, INF-*γ*, IL-2, IL-4, IL-6, IL-8, and TNF-*α* (pg/mL). The results are reported as the average of values for each cytokine assessed in every sample compared to the average of the cytokine levels in healthy fluids. Data presented by Tsuchida et al. (2014) [17] and Papalia et al. (2016) [26] and here presented to easily obtain a direct comparison. T-test analyses were performed between each pathological cytokine with respect to their healthy control (*∗*p<0.01) in addition to pathological IL-2 and IL-8 levels with respect to healthy IL-6 level (§p<0.01).

**Figure 4:** WB analysis of NF-kB and COMP-2 protein levels in chondrocytes (a) and synoviocytes. (b) Densitometric analysis of specifics bands obtained for NF-kB and COMP-2 expression has been normalized with respect to actin expression. Data shown are an average of two different western blotting with two densitometric recording each, reported as mean values ± SD. (a) Significant differences between H-HA and HCC versus P-CTRL and H-HA versus HCC are indicated with asterisks *∗*p<0.05, #p<0.01. Data shown are means ± SD. (b) Significant differences between H-HA and HCC versus P-CTRL and H-HA versus HCC are indicated with asterisks *∗*p<0.05, #p<0.01.

**Figure 5:** Analysis of IL-6, GM-CSF, IL-8, INF-*γ*, and TNF-*α* levels in supernatants (pg/mL) by the Bio-Plex cytokines assay of chondrocytes treated for 48 h with H-HA or HCC 0.32% w/v with respect to H-CTRL and P-CTRL. Data shown are means ± SD. Significant differences between H-HA and HCC versus P-CTRL, H-HA versus HCC, and H-HA or HCC versus H-CTRL are indicated with asterisks *∗*p<0.05, #p<0.01.

**Figure 6:** Human synoviocytes proliferation assay. (a) Pictures of cells at experimental times: 24, 48, 72, and 96 h; the proliferative properties of HCC were compared to the single H-HA and untreated synoviocytes (UT-S). (b) Cell growth curves were obtained through Image-Pro Plus 1.5 software (Media Cybernetics).

**Figure 7:** mRNA expression analysis of IL-6 and IL-8 in human synoviocytes isolated from osteoarthritic synovial fluid through qRT-PCR. (a) Quantitative gene expression of IL-6 and IL-8 in primary synoviocytes after 24 h of treatment with H-HA and HCC 0.32% w/v with respect to UT-S. (b) Gene expression of IL-6 and IL-8 in synoviocytes after 48 h of treatment with H-HA and HCC 0.32% w/v with respect to UT-S. Data shown are means ± SD. Significant differences between H-HA and HCC versus UT-S and H-HA versus HCC are indicated with asterisks *∗*p<0.05, #p<0.01.

**Table 1:** Primer sequences used for the qRT-PCR.

Gene	Forward Primer	Reverse Primer	AT PCR
GAPDH	5'-TGCACCACCAACTGCTTAGC-3'	5'- GGCATGGACTGTGGTCATGAG -3'	55°C
IL-6	5'- GTGGAGATTGTTGCCATCAACG -3'	5'- CAGTGGATGCAGGGATGATGTTCTG -3'	55°C
IL-8	5- ATGACTTCCAAGCTGGCCGT -3'	5'- TCCTTGGCAAAACTGCACCT -3'	55°C

## Data Availability

All data generated or analyzed during this study are included in this published article. All hyaluronan samples were kindly provided by Altergon s.r.l., Italy. Hybrid cooperative complexes were either obtained in our lab or diluted from Sinovial-HL syringes, commercialized by IBSA.

## Supplementary Materials

Supplementary Materials The supplementary files concerned FACS analyses relative to chondrocytes characterization (SF. Figure  1) using type II collagen as specific cartilage biomarker and synoviocytes cell (isolated by synovial fluid) characterization (SF. Figure  2) using different biomarkers. Specifically CD45+CD64+CD14+CD105+CD73+CD90±CD3-CD19-CD34- and CD105+CD73+CD90+CD45-CD64-CD14-CD3-CD19-CD34- were used to differentiate the two synoviocytes phenotypes: type A and type B.
